RETRACTED

# Enhancement of Lipid Productivity in Oleaginous *Colletotrichum* Fungus through Genetic Transformation Using the Yeast *CtDGAT2b* Gene under Model-Optimized Growth Condition

**DOI:** 10.1371/journal.pone.0111253

**Published:** 2014-11-06

**Authors:** Prabuddha Dey, Nikunj Mall, Atrayee Chattopadhyay, Monami Chakraborty, Mrinal K. Maiti

**Affiliations:** 1 Adv. Lab. for Plant Genetic Engineering, Advanced Technology Development Center, Indian Institute of Technology Kharagpur, Kharagpur, India; 2 Department of Biotechnology, Indian Institute of Technology Kharagpur, Kharagpur, India; Korea University, Republic of Korea

## Abstract

Oleaginous fungi are of special interest among microorganisms for the production of lipid feedstocks as they can be cultured on a variety of substrates, particularly waste lingocellulosic materials, and few fungal strains are reported to accumulate inherently higher neutral lipid than bacteria or microalgae. Previously, we have characterized an endophytic filamentous fungus *Colletotrichum* sp. DM06 that can produce total lipid ranging from 34% to 49% of its dry cell weight (DCW) upon growing with various carbon sources and nutrient-stress conditions. In the present study, we report on the genetic transformation of this fungal strain with the *CtDGAT2b* gene, which encodes for a catalytically efficient isozyme of type-2 diacylglycerol acyltransferase (DGAT) from oleaginous yeast *Candida troplicalis* SY005. Besides the increase in size of lipid bodies, total lipid titer by the transformed *Colletotrichum* (lipid content ∼73% DCW) was found to be ∼1.7-fold more than the wild type (lipid content ∼38% DCW) due to functional activity of the *CtDGAT2b* transgene when grown under standard condition of growth without imposition of any nutrient-stress. Analysis of lipid fractionation revealed that the neutral lipid titer in transformants increased up to 1.8-, 1.6- and 1.5-fold compared to the wild type when grown under standard, nitrogen stress and phosphorus stress conditions, respectively. Lipid titer of transformed cells was further increased to 1.7-fold following model-based optimization of culture conditions. Taken together, ∼2.9-fold higher lipid titer was achieved in *Colletotrichum* fungus due to overexpression of a rate-limiting crucial enzyme of lipid biosynthesis coupled with prediction-based bioprocess optimization.

## Introduction

Lipid is an important raw material for the production of different essential compounds related to food and non-food industrial applications. Among the food applications, storage lipid has been considered since many years as source of important fatty acids particularly polyunsaturated fatty acids (PUFAs) and other nutraceuticals as dietary supplements for fishes, poultry birds, domestic animals and human [1], [2]. Among non-food industrial applications, biodiesel production from lipid feedstock, specifically from plant seed oil, has massively increased recently. However, for sufficient production of oilseed crops fertile lands and several essential agro-inputs are required by plant. In addition to this, concerns about the global food security coupled with the increase in current food price and the competitive segregation of agricultural resources between the food industry and the energy sector have taken public awareness. Therefore, development of few sustainable and cost-effective alternatives to the traditional agricultural and forestry crops is of urgent need for biofuel production in the present scenario of escalating worldwide demand. Oil-rich microorganisms, specifically microalgae have been demonstrated to be a promising alternative source of lipids for biodiesel production [3], [4], [5]. There are several strains of bacteria, algae and fungi including yeasts and molds found in diverse natural ecosystems, which can accumulate storage lipid>20% of their dry cell weight (DCW), and are considered as oleaginous microbes. The important criteria for a microorganism to be acceptable for production of lipid feedstock are its total amount of lipid and the types of fatty acids inherently present in it.

RETRACTED

In last few years, production of microalgal lipid (also known as single cell oil) was primary research interest, but high amount of algal culture in industrial level either requires a large cultivation area or long incubation period in bioreactor system [6], which is also challenging due to necessity of appropriate light source [4]. Therefore, alternate oleaginous microbes, such as yeasts and filamentous fungi [6]–[8] are of special interest as they can be grown on a variety of starting materials (substrates), especially waste lignocellulosic materials; and biomass production can be scaled up in fermentation process to produce more total lipid. Filamentous fungi of Zygomycetes, like *Mortierella isabellina* and *Cunninghamella echinulata* have been reported with high amount of lipid content, i.e. 60–87% and 40–57% of DCW, respectively [9]. Our group has characterized two endophytic oleaginous fungi, *Colletotrichum* sp. DM06 and *Alternaria* sp. DM09, which can accumulate total lipid ∼34–58% of DCW during standard and nutrient stress conditions of growth; and the fatty acid profiles of their storage lipids are suitable for biodiesel application [10]. It is worthy to mention here that another oleaginous fungi *Mucor circnelloides* (having 20% lipid of DCW) has been used for the first commercial production of microbial lipid [1].

RETRACTED

From a long period of time, several strategies have been developed for overproduction of storage lipid in the selected microbial strain, besides bioprospecting of lipid hyper-accumulating novel isolate from natural resources. Among these, biochemical engineering approach that basically depends on creating a physiological stress such as nutrient-starvation (specifically nitrogen and phosphorous) to channel metabolic fluxes to lipid accumulation have been extensively carried out to enhance lipid accumulation in microorganism. The main requirement of fungi (i.e., molds and yeasts) for enhanced lipid production is the medium with excess carbon source and other limiting nutrients, mostly nitrogen [7], phosphorous [11], sulphur [12], aeration, inorganic salt, pH and temperature [13]. However, the biochemical engineering strategy (i.e., nutrient stress) limits the natural growth rate (cell division) of the organisms [1], [14], [9]. Since lipids are intracellular products, the overall lipid productivity is the product of cellular lipid content multiplied by total biomass titer. Hence, the overall lipid titer will be compromised due to the lower biomass productivity. Therefore to overcome this bottleneck, scientists have devised genetic or metabolic engineering approach.

In the past three decades, metabolic engineering strategies by overexpressing or down-regulating several important rate-limiting enzymes to create a channeling of metabolites towards lipid accumulation in different plant and microbial species have already been carried out. Many of the genes, like *ACC1*, *DGAT*, *LPAT*, *malE*, *ACL* and *PEPC* [15] involved in the lipid metabolism have been subjected to be overexpressed [16] and or silenced in oleaginous seeds of higher plant [17]–[20], bacteria [21], yeast [18], fungus [22] and algae [23]; and these genetic modifications have resulted in increased production of fatty acids and storage lipids or triacylglycerol (TAGs). In microbial systems, the most promising targets are diacylglycerol acyltransferase (DGAT) and malic enzyme (ME) for gene overexpression, and phosphoenolpyruvate carboxylase (PEPC) is for down-regulation in order to enhance storage lipid productivity [24]. The DGAT enzyme catalyzes the final step of TAG biosynthesis in most of the TAG-accumulating cells/organisms by transferring an acyl group from acyl-CoA to the sn-3 position of 1,2-diacylglycerol. The success with overexpression of DGAT could be explained by the fact that the substrate of DGAT i.e., diacylglycerol, naturally could be allocated to either phospholipid biosynthesis or TAG biosynthesis. Overexpression of DGAT would commit more diacylglycerol to TAG formation rather than phospholipid formation. The *DGAT* gene has been transgenically overexpressed in yeast and plant systems to enhance storage lipid production [18], [20], [25], [26]. However, no report regarding the overexpression of this crucial enzyme in filamentous fungi was available in published literatures till the present study.

RETRACTED

Model-based bioprocess optimization of media condition is one of the most important tools for obtaining increased yield of any fermentative product. The most effective method is the statistical approach to evaluate the relative significance of the variables in the medium for optimization of target metabolite production. Different statistical method like Plackett–Burman, response surface methodology (RSM) and factorial designs have been used in past few decades for optimization of medium. A mathematical approach such as artificial neural network (ANN) coupled to genetic algorithm (GA) is recently gaining popularity and found to be superior to other statistical approach like, RSM [27], [28].

As already mentioned, the endophytic filamentous fungus *Colletotrichum* sp. DM06, which we have isolated, can accumulate>34% DCW and>49% DCW of total lipid without and with nutrient stress condition, respectively [10]. Moreover, our group has also recently characterized two structurally novel type-2 DGAT isozymes, CtDGAT2a and CtDGAT2b from an oleaginous rhizospheric yeast *Candida tropicalis* SY005 [29], and documented that the CtDGAT2b is catalytically 12.5% more efficient than CtDGAT2a for TAG production [30]. Therefore, in the present study we aimed to overexpress the more efficient CtDGAT2b isozyme of *C. tropicalis* in *Colletotrichum* fungus to increase the production of storage lipid. Another objective of this study was to establish the optimum culture conditions (with respect to temperature, pH, carbon: nitrogen and carbon: phosphorous ratio of growth medium) through model-based prediction so as to further increase the lipid productivity in the genetically modified *Colletotrichum* strain.

## Materials and Methods

### Strain, media and growth condition

*Colletotrichum* sp. DM06 strain, an endophytic wild type fungus isolated from the medicinal plant *Ocimum sanctum* [10], was cultured on potato dextrose agar (PDA) medium at 28°C. The composition of the basal liquid medium for lipid production has been described previously [10]. *Escherichia coli* strain DH10B was used for maintainance of binary plasmid and cultivated at 37°C on LB agar plates or liquid medium containing 50 µg/ml kanamycin. *Agrobacterium tumefaciens* LBA4404 was used as a transfer DNA (T-DNA) donor for fungal transformation. YEP medium (consisting of 10 g/l yeast extracts, 10 g/l peptone and 5 g/l NaCl) was used for cultivation of *A. tumefaciens* LBA4404 at 28°C.

RETRACTED

### Preparation of genetic constructs

The pCAM-GpdA-GusA-TrpC genetic construct was prepared using the backbone of pCAMBIA 1300 binary vector. Initially the pNOM102 vector carrying the intron-containing *gusA* (*uidA*) gene placed under the regulation of *gpdA* promoter of *Aspergillus nidulans* and *trpC* terminator of *A. nidulans* in pUC18 vector (kindly provided by Prof. Francisco JL Aragão, Embrapa Recursos Genéticos e Biotecnologia, Brazil) was doubly digested with *Eco*RI and *Hind*III to obtain the DNA fragment GpdA-GusA-TrpC, which was subcloned into the pCAMBIA 1300 using the same set of restriction enzymes. The resulting recombinant plasmid was named as pCAM-GpdA-GusA-TrpC (Figure 1A). Cloning, sequencing and characterization of the *CtDGAT2b* gene (GenBank accession number KJ437598) from *Candida tropicalis* SY005 have already been described previously [30]. The *CtDGAT2b* gene was obtained after digesting with *Bam*HI from pYES2/CtDGAT2b recombinant plasmid, which was used for the study of transgene expression in *Saccharomyces cerevisiae* [30]. The promoter GpdA was PCR amplified from pCAM-GpdA-GusA-TrpC recombinant plasmid (using Expand High Fidelity PCR mix, Roche) with a set of specific primers- GpdAFp and GpdARp (Table S1) to incorporate the restriction sites- *Eco*RI at 5' end and *Bam*HI at 3' end of the promoter. The pCAM-GpdA-GusA-TrpC construct was digested with *Eco*RI and *Bam*HI to remove the GpdA promoter and *gusA* gene. Thereafter, a tripartaite ligation was carried out using the *Bam*HI digested *CtDGAT2b* gene, *Eco*RI and *Bam*HI digested PCR amplified GpdA promoter and the above-mentioned *Eco*RI and *Bam*HI digested pCAM-GpdA-GusA-TrpC to generate the pCAM-GpdA-CtDGAT2b-TrpC recombinant plasmid (Figure 2A).

**Figure 1:** Standardization of *Agrobacterium*-mediated transformation of *Colletotrichum* fungus with the *gusA* reporter gene expression construct, pCAM-GpdA-GusA-TrpC. (A) Schematic diagram of the genetic construct prepared in pCAMBIA1300 binary vector. (B) Ethidium bromide-stained 1.2% agarose gel showing characteristic restriction enzyme digestion profile of the genetic construct with *Xho*HI (lane 1), *Eco*RI+*Hind*III (lane 2), *Eco*RI+*Sal*I (lane 3), *Eco*RI+*Bam*HI (lane 4) and *Bam*HI+*Hind*III (lane 5) along with the pUC18 DNA digested with *Hin*f1 as molecular weight marker (lane 6). (C) PCR-based screening for the presence of 450 bp *hptII* selection marker gene-specific amplicon in four (Tg#1, Tg#4, Tg#7 and Tg#13) chosen transformed lines. (D) PCR-based screening for the presence of 1100 bp *gusA* reporter gene-specific amplicon in the same four transformed lines. In (C) and (D), Lane M =  *Hin*fI digested pUC18 DNA as molecular weight marker (E) Confirming genomic integration of the *gusA* transgene through Southern hybridization. Genomic DNA samples of three (Tg#4, Tg#7 and Tg#13) transformed lines were digested with *Eco*R1 (lane E) and *Hin*dIII (lane H) seperately, and hybridized with the *gusA* gene-specific probe. Lambda (λ) DNA digested with *Eco*RI+*Hind*III was used as molecular weight marker. In case of (C), (D) and (E), the wild type *Colletotrichum* sp. DM06 was taken as control (lane C). (F) Histochemical GUS assay in fungal transformant Tg#4 depicting functional activity of the *gusA* transgene along with the wild type strain as control. Microscopic visualization of GUS activity in different fungal tissues at variable magnifications: mycelium at 10X (1), hypha at 100X (2), spores at 1000X (3) and setae at 40X(4).

RETRACTED

**Figure 2:** Development of *Colletotrichum* transformants with the *CtDGAT2b* gene expression construct, pCAM-GpdA-CtDGAT2b-TrpC through *Agrobacterium*-mediated transformation. (A) Schematic diagram of the genetic construct prepared in pCAMBIA 1300 binary vector. (B) Ethidium bromide-stained 1.2% agarose gel showing characteristic restriction enzyme digestion profile of the genetic construct with *Eco*RI+*Hind*III (lane1), *Eco*RI+*Bam*HI (lane2), *Bam*HI (lane3), *Sal*I+*Bgl*II (lane 4), *Bam*HI+*Hind*III (lane 5) and *Xho*HI (lane 7) along with the pUC18 DNA digested with *Hin*f1 as molecular weight marker (lane 6). (C) PCR-based screening for the presence of 550 bp *CtDGAT2b* transgene-specific amplicon in four (Td#2, Td#9, Td#18 and Td#23) chosen transformed lines. Lane M =  *Hin*fI digested pUC18 DNA as molecular weight marker. (D) Confirming genomic integration of the *CtDGAT2b* transgene through Southern hybridization. Genomic DNA samples of four transformed lines were digested with *Eco*R1, and hybridized with the *CtDGAT2b* gene-specific probe. Lambda (λ) DNA digested with *Eco*RI+*Hind*III was used as molecular weight marker. In case of (C) and (D), the wild type *Colletotrichum* sp. DM06 was taken as control (lane C). (E) Transcriptional expression of the *CtDGAT2b* transgene in four fungal transformants as revealed by RT-PCR for 26 cycles. (F) Transcriptional expression of the *CtDGAT2b* in one of the fungal transformants, Td#18 (T) as revealed by RT-PCR for 26 cycles, showing upregulation of CtDGAT2b transcript upto 3^rd^ day of growth and declined at 4^th^ day onward. In case of (E) and (F), the wild type *Colletotrichum* sp. DM06 was taken as control (C), and the relative transcript level was measured based upon the densitometric scanning of the RT-PCR amplicons (550 bp for *CtDGAT2b* and 400 bp for endogenous *β-actin* as internal control) as shown in lower panel.

RETRACTED

### Agrobacterium tumefaciens-mediated transformation of Colletotrichum fungus

Prior to perform the *A. tumefaciens*-mediated transformation (ATMT), the antibiotic susceptibility test of wild type *Colletotrichum* sp. DM06 was carried out on hygromycin B (used as the selection marker for the transformants). Results showed that a dose of 200 µg/ml of hygromycin B completely inhibited the growth of wild type fungus (data not shown), therefore this concentration of antibiotic was used for the selection of fungal transformants.

ATMT was carried out following the method described earlier [31] with certain modification. An aliquot of 10% (v/v) of *Colletotrichum* sp. DM06 spore maintained in glycerol stock was spread on PDA plates and incubated at 30°C for 4 days for sporulation. Spores were collected, washed and suspended in induction media (IM) [32], and adjusted to a concentration of 10^3^-10^6^ conidia/ml. *A. tumefaciens* LBA4404 strain carrying the desired genetic construct was initially grown on YEP media supplemented with 20 µg/ml rifampicin, 75 µg/ml chloramphenicol and 50 µg/ml kanamycin at 28°C with shaking at 250 rpm for 24 h. Next day, 1.5 ml of *Agrobacterium* culture was pelleted down, washed and resuspended in IM either in absence or presence of 0.2 M acetosyrengone (AS), and allowed to grow until it reached OD_600_∼ 0.8. One hundred microliter of the induced *Agrobacterium* cells and 100 µl of the fungal conidiospores were mixed. This 200 µl mixture was pipetted and spread evenly onto sterile nitrocellulose membrane (diameter 130 mm) placed over the solid IM with or without AS. Keeping the bacterial suspension constant, variable concentrations of the conidial suspension were tested (ranging from 10^2^ to 10^5^ conidia per plate). Different temperature (20°C to 25°C) and duration (2 to 5 days) of co-cultivation were tested to find out optimum condition of transformation for this fungal strain. After co-cultivation of the plates, the membranes containing the *Agrobacterium*–fungal mixture were removed and placed on PDA plates containing hygromycin B 200µg/ml. The plates were incubated at 28°C until transformed fungal colonies appeared. After obtaining some putative fungal transformants they were maintained on PDA media containing hygromycin. The stability of the randomly selected transformants was tested at least five times on fresh medium with or without hygromycin.

### PCR-based screening and Southern hybridization of the transgene in fungal transformants

Screening of putative fungal transformants was carried out among several hygromycin positive clones by PCR using *gusA* or *CtDGAT2b* transgene-specific set of primers (Table S1). For Southern hybridization, 10 µg of genomic DNA from the wild type control fungus and from randomly selected few stable transformants were digested with restriction enzymes and size-fractionated on 0.8% agarose gel along with DNA molecular weight marker. Transfer of nucleic acids onto nylon membrane and hybridizations with [α−^32^P]dCTP labeled transgene-specific probe were performed following standard techniques [33].

RETRACTED

### Histochemical GUS assay

Histochemical GUS assay of the stable fungal transformants was carried out following standard procedure [34]. Fresh mycelia were submerged in GUS assay buffer (0.1 M sodium phosphate buffer, pH 7.0, 0.1% Triton X-100 and 2 mM X-Gluc) and incubated at 37°C for ∼8–10 h in order to develop the characteristic blue color. Following that, mycelia were washed with 70% ethanol and stored in 70% ethanol till photography.

### Total RNA extraction and semi-quantitative RT-PCR

Total RNA was extracted from the wild type and fungal transformants using RNA extraction kit (RNeasy plant mini kit, Qiagen, India) according to the manufacturer's protocol. RNA quantity was measured by spectrophotometric reading at 260/280 nm, and the quality of RNA was determined by observing the integrity of rRNA bands in 1.2% agarose gel. For RT-PCR analysis, a set of specific primers was designed (Table S1). The 1^st^ strand cDNA was synthesized by respective gene-specific reverse primers with the High-Capacity cDNA Reverse Transcription Kits (Applied Biosystems) using 3 µg total RNA as template according to the manufacturer's protocol. The products of RT-PCR were subjected to electrophoresis in 1.5% agarose gel and visualized under UV trans-illuminator following ethidium bromide staining.

### Microscopy following Nile red staining

The Nile red is a lipid-specific dye. Confocal microscopic analyses of the Nile red-stained wild-type and transformed fungal cells were carried out to examine the presence of storage lipid bodies in mycelia as described previously [35] with certain modification [10]. The samples were observed under laser-scanning confocal microscope with 488 nm excitation and 585 nm emission filters (Fluo View FV1000 confocal microscope, Olympus).

### Lipid extraction and fractionation

For extraction of total lipid from the wild-type and transformed fungal biomass, normal chloroform: methanol extraction procedure was followed, and estimation was carried out following Bligh and Dyer method [36] with slight modification as described earlier [10]. Total lipid was fractionated into neutral lipid and estimated using a silica cartridge (Sep-Pak Vac 6cc, Waters) following the method described earlier [10]. Both the quantitative estimations of total lipid and neutral lipid were conducted with three individual cultures for each set of experiments and with three replicates.

RETRACTED

### Preparation of fatty acid methyl esters and determination of fatty acid profiles

Fatty acid methyl ester (FAME) of the total lipid fraction from the wild type and transformed fungal cells was prepared following the method described earlier [10]. Finally, small volume (3-5µl) of the prepared FAME sample was analyzed by gas chromatography (GC) instrument (Clarus 500, PerkinElmer), fitted with a flame ionization detector (FID) and Omegawax-250 capillary column (30 m length, 0.25 mm internal diameter and 0.25 µm film thickness, Sigma). Identification and quantification of individual chromatographic peaks were carried out by means of external standard (Supelco 37-Component FAME Mix, Sigma) and their corresponding calibration curves. Samples were taken from three individual cultures for each set of experiments and with three replicates.

## Results

### Standardization of *Agrobacterium*-mediated transformation of *Colletotrichum* sp. DM06 strain using *gusA* reporter gene construct

Genetic transformation of *Colletotrichum* sp. DM06 was standardized using *Agrobacterium tumefaciens* LBA4404 strain harboring the *gusA* reporter gene construct pCAM-GpdA-GusA-TrpC (Figure 1A). Analysis of the restriction enzyme digestion profile of the recombinant plasmid confirmed the correct orientation of the genetic elements (Figure 1B). Prior to start of transformation the antibiotic susceptibility test of wild type *Colletotrichum* sp. DM06 was carried out on hygromycin B to be used as the selection marker for the transformants. Results showed that hygromycin concentration of 150 µg/ml inhibited the growth of wild type *Colletotrichum* sp. DM06 extremely, whereas the growth was completely inhibited at 200 µg/ml (data not shown). Therefore, a dose of 200 µg/ml of hygromycin B was used for the selection of transformants during *Agrobacterium*-mediated transformation of *Colletotrichum* sp.

After collecting the fungal spores (conidia), initial step of transformation was performed by spreading a mixed suspension of fungal spores and *Agrobacterium* cells on sterile nitrocellulose membranes placed on agar plates without or with acetosyringone (AS), which is necessary for the induction of *vir* genes, followed by successive incubation for cocultivation. Temperature, duration and concentration of *Agrobacterium* cells for cocultivation were optimized for this particular fungal strain. The optimum temperature for cocultivation was found to be 23°C for a period of 3 days at 0.6 cell density (OD_600_) of *A. tumefaciens* cells. Further incubation for a prolonged period of 5 days increased excessive mycelial growth of *Colletotrichum*, which created difficulties in isolation of individual transformants in AS containing plates. Similar result was obtained with the increased number of *Agrobacterium* cells as well.

RETRACTED

After cocultivation for 3 days at 23°C, the nitrocellulose membrane was transferred to hygromycin (200 µg/ml) containing plate, and incubated for 5 days at 28°C until putative transformants were visible. We could usually obtain 40 to 100 transformants per 5×10^5^ numbers of conidia of *Colletotrichum* sp. DM06. Transformation with more number of conidia (1×10^6^) produced a mycelial lawn, which made it complicated to isolate individual transformant (data not shown). Moreover, incubation of *Agrobacterium* cells with AS prior to cocultivation, and addition of AS to plates during cocultivation enhanced the number of putative transformants than the AS negetive plates (data not shown).

### Analysis of the fungal transformants for inheritance stability, genomic integration and functional expression of the transgene

The inheritance stability of the hygromycin resistant gene in putative transformants was examined by transferring mycelia from the edge of transformed colonies at least five times to new medium with and without hygromycin. Among the 40 transformants obtained, 15 were adjudged as stable, whereas other lost the hygromycin resistant phenotype after serial subculture on antibiotic selective medium. Among the 15 stable transformants, four (Tg#1, Tg#4, Tg#7 and Tg#13) were selected for further analyses because these four were significantly more stable, retaining their ability to grow rapidly on hygromycin selective medium after five serial subcultures on non-selective medium.

Verification of the transgene integration onto the fungal genome was carried out by PCR using two gene-specific primer pairs (Table S1) and subsequently confirmed by Southern hybridization. The presence of amplified fragments of 450 bp (Figure 1C) and 1100 bp (Figure 1D) in genomic DNA samples from transformed colonies revealed the existence of the *hptII* and *gusA* transgenes, respectively. The genomic DNA sample from the non-transformed colony did not show any PCR-amplified fragment specific for these two transgenes (Figure 1C, 1D). To confirm the integration and copy number of the transgene in the respective genomes of selected *Colletotrichum* transformants, Southern blot analysis was performed using genomic DNA samples isolated from the PCR-positive and non-transformed fungal colonies. Genomic DNA samples were digested with *Eco*R1 and *Hin*dIII seperately, and hybridized with the *gusA* gene-specific probe. All the three transformant lines tested (Tg#4, Tg#7 and Tg#13)) showed clear hybridization signal for transgene integration onto the corresponding genomes (Figure 1E). Genomic DNA from the non-transformed colony was used as a negative control and showed no hybridization signal (Figure 1E). The T-DNA region of the pCAM-GpdA-GusA-TrpC (Figure 1A) recombinant plasmid has only one *Hin*dIII and *Eco*RI site each. In transformed fungal colony Tg#7, two hybridization signals for *Eco*R1 and *Hin*dIII indicated two copies of T-DNA integration in this line (Figure 1E), while transformant Tg#13 showed three hybridization signals for both the enzymes indicating that three copies of T-DNA integrated onto the genome of this transformed line (Figure 1E). On the contrary, single hybridization signal for both the enzymes in transformed line Tg#4 specified one copy of transgene integration in this fungal genome (Figure 1E).

RETRACTED

Functional expressions of the transgene in selected transformants were verified by histochemical GUS assay. A high percentage GUS positive cells were detected in the transformed mycelia, indicating successful expression and functional activity of the *gusA* gene. Characteristic blue staining was visible within the fungal hyphae, conidia and setae of Southern- positive fungal transformants through microscopic examination, as shown for Tg#4, one of the transformed lines (Figure 1F).

### Generation of *Colletotrichum* transformants using *CtDGAT2b* gene construct

*A. tumefaciens* LBA4404 strain harbouring the recombinant plasmid pCAM-GpdA-CtDGAT2b-TrpC (Figure 2A) that contains the target gene *CtDGAT2b* was used to genetically transform the *Colletotricum* sp. DM06 following the transformation protocol standardized using the *gusA* reporter gene construct. Restriction enzyme digestion of the recombinant plasmid was carried out before transformation to confirm the correct orientation of different genetic elements including the *CtDGAT2b* gene (Figure 2B). Putative fungal transformants harbouring the *CtDGAT2b* gene were selected on hygromycin (200µg/ml) plate, as performed for *gusA* gene transformation. Few selected putative *Colletotrichum* transformants (Td#2, Td#9, Td#18 and Td#23) showing effective growth on both antibiotic selective and non-selective media after 5 cycles of subculture, were subjected to PCR screening using *CtDGAT2b* gene-specific primer pair (Table S1). An expected size 550 bp amplicon specific for *CtDGAT2b* gene was revealed in all four selected transformants, but no such amplified product was detected in untransformed control colony (Figure 2C). To confirm the integration of transgene in the fungal genome, Southern hybridization of the *Eco*RI digested genomic DNA isolated from each of the PCR-positive transformants along with untransformed fungal cells was carried out using the *CtDGAT2b* gene-specific probe (Figure 2D). Among the four PCR-positive transformants tested, Td#2 and Td#23 showed single copy genomic integration of the transgene, whereas two copies of transgene were found to be integrated into the genome of Td#9 and Td#18 transformsnts. On the contrary, no such Southern hybridization signal was observed for the untransformed control (Figure 2D). Further qualitative and quantitative analyses of storage lipid were carried out in these four stable transformants after examining the transgene expression.

RETRACTED

To verify the expression of *CtDGAT2b* transgene in *Colletotrichum* transformants, semi-quantitative RT-PCR was carried out using the DNaseI-treated total RNA samples isolated from Southern-positive transformants along with the untransformed fungal cells. Under the conditions described in the methods, the exponential phase of RT-PCR using CtDGAT2b-specific primers was detected between 24 to 28 cycles (data not shown). Subsequently, the RT-PCR for 26 cycles yielded a 550 bp *CtDGAT2b*-specific amplicon in all the samples of fungal transformants, whereas no such RT-PCR amplicon was obtained in untransformed control (Figure 2E). No DNA fragment was PCR-amplified by transgene-specific primer set using the DNaseI-treated total RNA samples directly as the templates (without reverse transcription), indicating absence of genomic DNA contamination in the RNA samples used for RT-PCR (data not shown). When quantitative variations of the *β-actin* transcript were correlated with that of the *CtDGAT2b* transcript, a slightly enhanced expression level of *CtDGAT2b* transgene was observed in the fungal transformant till certain time periods of growth, as depicted for Td#18, one of the transformants (Figure 2F). A clear upregulation of the *CtDGAT2b* transcript was recorded at 3^rd^ day of growth, and its expression declined at 4^th^ day onward.

### Enhanced accumulation of storage lipid with altered fatty acid profile in transformed fungal cells expressing *CtDGAT2b* transgene

Fungal mycelia from both the transformant and nontransformant were stained with lipid-specific Nile red dye, and visualized by confocal microscopy. Significant increase in fluorescence intensity was observed in the transformant with *CtDGAT2b* transgene compared to the control fungal cells at different magnification of microscopy (Figure 3A). Moreover, an average increase in size of lipid droplets was noticable throughout the transformed mycelia on comparision to nontransformant at 60X magnification (Panel 4, Figure 3A). This result revealed that CtDGAT2b transformed fungal cells accumulated higher amount of storage lipid compared to the nontransformant. Quantitative details of the total lipid and neutral lipid production in four stable transformants are presented in the next subsection. Fatty acid profiles of the four stable transformants expressing the *CtDGAT2b* gene along with the untransformed fungal cells were examined through GC-FID of FAME samples prepared from total lipid. Analysis revealed that the contents of saturated fatty acids, particularly palmitic acid (C16:0) and stearic acid (C18:0), were found to be increased, but the amount of oleic acid (C18:1) decreased in all four transformants compared to the untransformed fungus (Figure 3B). The contents of C16:0 and C18:0 in transformants were approximately 30–58% and 40–58% more, respectively compared to the wild type; whereas the C18:1 content of the transformants was about 28–35% less with respect to wild type.

RETRACTED

**Figure 3:** Alteration in the quality and quantity of storage lipid due to functional activity of CtDGAT2b in *Colletotricum* transformants. (A) Nile red stained confocal microscopic images of mycelia of the wild-type (control) and one of the transformed lines (Transformant). Panels 1 to 4 represent microscopic images of mycelia at different magnifications, and each panel has identical scale bar for both the control and transformant. In panels 1 and 2, scale bar  = 10 µm showing same magnification but at different location of mycelia. In panels 3 and 4, scale bar  = 5 µm and 2 µm, respectively. White arrow indicates increase in size of lipid droplets in mycelia of transformant. (B) Bar diagram representing fatty acid profile (relative % of fatty acids) in total lipid samples obtained from the wild-type and four transformants as revealed by GC-FID analysis. (C) Bar diagram showing total lipid content expressed as % of dry cell weight (% DCW) during standard growth condition (black bar), nitrogen starvation (white bar) and phosphorus starvation (grey bar) among the wild type control (C) and four (Td#2, Td#9, Td#18 and Td#23) fungal transformants. (D) Bar diagram depicting neutral lipid content expressed as % of total lipid content during above-mentioned three growth conditions among the wild type control (C) and the same four fungal transformants.

### Functional expression of *CtDGAT2b* increases lipid titer in transformed *Colletotrichum* lines upon both standard and stress conditions of growth

Detailed estimation of the lipid productivity was carried out to determine the differences between the wild type and the transformed *Colletotrichum* lines, in order to analyze the effect of expressing yeast *CtDGAT2b* gene in fungal cells. Our previous study indicated that in high glucose-containing media, nitrogen and phosphorus are the limiting nutrient factors for lipid titer in this endophytic fungus [10]. Therefore, three culturing conditions were evaluated in the present study to find out *in vivo* effect of target gene overexpression: (i) standard condition (i.e., nutrient repleat condition), (ii) nitrogen stress condition and (iii) phosphorus stress condition.

RETRACTED

Four stable transformants along with the wild type *Colletotrichum* sp. DM06 were cultured in the three above-mentioned conditions of growth, and total lipid was extracted and estimated from cell biomass of each sample. In standard condition (i.e., without nutrient stress) the wild type fungus produced about 4.8±0.1 g/l of total lipid that corresponds to 38.4±0.4% of dry cell weight (DCW), whereas in similar condition the four stable transformants produced on an average 8.1±0.2 g/l of total lipid ( = 73.6±0.6% DCW) (Table 1, Figure 3C). Thus, the lipid titer of transformed cells was ∼1.7-fold higher than the wild type strain at standard growth condition, indicating an increase of lipid content by ∼92% DCW. Moreover, when tested in nitrogen stress (C:N 160:1) and phosphorus stress (C:P 86:1) conditions (previously standardized as optimum conditions for highest lipid titer of this fungus, [10]); the wild type fungus produced total lipid around 7.7±0.2 g/l ( =  42.5±0.1% of DCW) and 7.9±0.4 g/l of total lipid ( = 42.8±0.4% of DCW), respectively (Table 1, Figure 3C). In comparision to these data, the four stable transformants produced an average 12.2±0.7 g/l ( = 75.2±0.4% DCW) and 12.1±0.1 g/l ( = 75.2±0.4% DCW) of total lipid in nitrogen and phosphorus stress conditions, respectively (Table 1, Figure 3C). Therefore, the lipid titer of transformed cells was ∼1.5-fold more than the wild type fungus in stress conditions of growth, implying an enhancement of lipid content by ∼78% DCW.

**Table 1:** Estimation of biomass titer (g/l), total lipid titer (g/l), total lipid content (%DCW), neutral lipid titer (g/l) and neutral lipid content (% total lipid content) from cultures of wild type and transformed *Colletotrichum* cells grown in three different conditions for 10 days.

Conditions of growth	Organism	Biomass titer (g/l)	Total lipid titer (g/l)	Total lipid content (%DCW)	Neutral lipid titer (g/l)	Neutral lipid content (%DCW)
**Standard**	Wild-type	12.5±0.4	4.8±0.1	38.4±0.4	2.2± 0.7	17.6 ± 0.8
	Transformant^a^	11±0.6	8.1±0.2	73.6±0.6	4.0± 0.8	36.3± 0.6
**Nitrogen stress**	Wild-type	18.2±0.8	7.7±0.2	42.5±0.1	3.6± 0.7	19.7 ± 0.6
	Transformant^a^	16.2±0.1	12.2±0.7	75.2±0.4	6.1 ± 0.8	37.6 ± 0.6
**Phosphorus stress**	Wild-type	18.5±0.5	7.9±0.4	42.8±0.4	4.3 ± 0.4	23.2 ± 0.3
	Transformant^a^	16.2±0.5	12.1±0.1	75.2±0.4	7.1 ± 0.3	43.8 ± 0.8

a =  average value for four stable transformed lines- Td#2, Td#9, Td#18 and Td#23

To examine whether the heterologous expression of *CtDGAT2b* gene directly influences the neutral lipid production in fungal transformants, the total lipid of each sample was fractionated to recover neutral lipid component for its measurement. The wild type fungus produced neutral lipid ∼2.2±0.7 g/l ( = 17.6±0.8% DCW) in standard condition, ∼3.6±0.7 g/l ( = 19.7±0.6% DCW) in nitrogen stress condition, and ∼4.3±0.4g/l ( = 23.2±0.3% DCW) in phosphorus stress condition (Table 1, Figure 3D). On the contrary, the four transformants produced an average ∼4.0±0.8 g/l ( = 36.3±0.6% DCW), ∼6.1±0.8 g/l ( = 37.6±0.6% DCW) and 7.1±0.3 g/l ( = 43.8±0.8% DCW) of neutral lipid in standard, nitrogen and phosphorus stress conditions, respectively (Table 1, Figure 3D). Taken together, it was observed that the neutral lipid titer in transformants increased upto 1.8-fold, 1.6-fold and 1.5-fold compared to the wild type when grown under standard, nitrogen stress and phosphorus stress conditions, respectively. From these findings it could be inferred that the *CtDGAT2b* gene has been successfully utilized for enhanced neutral lipid production in transformed *Colletotricum* lines.

RETRACTED

### Model-based optimization of culture conditions to maximize lipid productivity in transformed *Colletotrichum* cells

The four critical parameters influencing lipid productivity of *Colletotrichum* fungus i.e., temperature, pH, carbon: nitrogen ratio and carbon: phosphorus ratio as revealed by our previous study [10] were taken into account to find out the optimum conditions for lipid production in transformed fungal cells. The central composite design (CCD) ensured statistically well distributed 30 data points for modelling using artificial neutral network (ANN) based on these four growth parameters (Table S2). After estimation of biomass titer and total lipid titer of the wild type (Table S3, S5) and one (Td#2) of the transformants (Table S4, S6) grown in 30 different conditions, the optimum growth conditions for maximum lipid accumulation were set up (Table 2). The regression correlation coefficient between the ANN-simulated values and actual experimental values of lipid titer was 0.97724 for wild type and 0.98541 for transformed organism (Table S7). The Mean Squared Error (MSE) and Mean Absolute Error (MAE) of predicted lipid yield for wild type fungus were 0.0174 and 0.0118, respectively; whereas the MSE and MAE of predicted lipid titer for transformed fungus were 0.0161 and 0.0130, respectively (data not shown). Genetic algorithm was run for a maximum of 500 iterations to observe a gradual convergence of the best fitness values of successive generations giving the optima for both the strains. Once we have the optimum conditions of lipid accumulation for both wild type and transformant seperately, it was easier to compare the lipid accumulating ability among them. The experimental result showed that the highest lipid titer in best optimum condition for the wild type fungus was 9.1±0.8 g/l, whereas for the transformant it was 14.1±0.5 g/l (Table 3). We cross-validated the optimal conditions by switching the wild type strain under the transformant's optimal conditions, and the transformant under the wild type's optimal conditions. Analysis of the data revealed that switching the optimal condition for growth did not alter lipid content significantly (Table 3). Therefore, the lipid titer of transformed cells was ∼1.5-fold greater than the wild type strain in model-optimized growth condition, indicating an increase of lipid content by ∼73% DCW.

RETRACTED

**Table 2:** Predicted biomass titer, lipid titer and lipid content in the wild type and transformed fungal cells through model-based optimization of growth conditions

Organism	Temperature	pH	C:N	C:P	Predicted biomass titer (g/l)	Predicted lipid titer (g/l)	Predicted lipid content (%DCW)
**Wild type**	27.3	6.30	129.46	83.32	18.2	9.5	52.8
**Transformant**	29.6	6.61	152.07	108.08	17.5	14.74	86.7

**Table 3:** Experimentally determined values of biomass titer, lipid titer and lipid content in the wild type and transformed fungal cells cultured in model-optimized growth conditions.

Organism	Temperature	pH	C:N	C:P	Experimental biomass titer (g/l)	Experimental lipid titer (g/l)	Experimental lipid content (%DCW)
**Wild type**	27	6.3	129	83	18.5±0.7	9.1±0.8	49.2±0.6
**Transformant**	27	6.3	129	83	15.5±0.4	12.4±0.5	79.2±0.4
**Wild type**	29	6.6	152	108	17.6±0.5	8.4±0.6	47.5±0.6
**Transformant**	29	6.6	152	108	16.2±0.9	14.1±0.5	85.4±0.3

## Discussion

Previously, we have characterized an endophytic fungus *Colletotrichum* sp. DM06, which is capable of accumulating significant amount of storage lipid having biodiesel properties [10]. This *Colletotrichum* strain can produce high amount of total lipid (∼7.8±0.2 g/l) using simple sugar, and substantial quantity of total lipid (∼84.3±3.9 mg/gds) utilizing lignocellulosic substrates that are degraded by the inherent secretory enzymes including cellulase. The results of both liquid culture and soild state fermentation for lipid production are promising and provided clue for further investigation towards strain improvement of this filamentous fungus to produce lipid feedstock in cost-effective way. Therefore, we have adopted the genetic engineering strategy to overexpress a critical rate-limiting enzyme involved in lipid biosynthesis along with the prediction-based optimization of culture conditions. The *CtDGAT2b* gene (encoding for a type-2 DGAT isoform from the oleaginous yeast *C. tropicalis*) has been transgenically introduced in *Colletotrichum* sp. DM06 to increase the metabolic flux towards the production of storage lipid in the transformed fungus. Additionally, ANN-based optimization of culture conditions (with respect to temperature, pH, carbon: nitrogen ratio and carbon: phosphorus ratio) has been established to further enhance the lipid productivity in the genetically improved *Colletotrichum* strain.

RETRACTED

*Agrabacterium tumefacience*-mediated transformation (ATMT) in fungus is already in practice by scientists to genetically improve the strain for the production of desired metabolite, but the protocol varries among fungal genera. Generally, the most commonly used antibiotic selection agent for fungal transformants is hygromycin B, and the dose is 100 µg/ml [37], [38]. However, there are previous reports on few species of *Colletotrichum* genus, where hygromycin sensitivity of 50 µg/ml to 300 µg/ml has been recorded [39]. Similar to different plant species, as various fungal strains of same genus have species-specific sensitivity on hygromycin; here firstly we have tested the antibiotic sensitivity dose on wild type isolate *Colletotrichum* sp. DM06, and finally 200 µg/ml concentration of hygromycin B was used for the selection of genetic transformants. Previous study showed that the effectiveness of transformation could be increased in presence of AS for different fungal species [40]. Moreover, few studies reported that the efficiency of fungal transformation is dependent primarily on the temperature, cocultivation duration, and concentration of the bacterial cell suspension [41], [37], [42], [39]. In a variety of Ascomycetes fungi, generally 10^6^ numbers of conidia have been used for ATMT experiment [41]. In the present study, we have standardized the ATMT of *Colletotrichum* sp. DM06 strain with *gusA* reporter gene, and it was found that cocultivation of 5×10^5^ numbers of fungal conidia with 0.8 cell density (OD_600_) of *A. tumefacience* (LBA4404) cells at 23°C for 3 days and incubation with AS were optimum. After confirmation of the inheritance stability and genomic integration of the transgene in few transformed lines, phenotypic expression of the transgene was validated in selected fungal transformants through histochemical GUS assay.

RETRACTED

In order to improve the production of storage lipid (TAG) in *Colletotrichum* sp. DM06 strain, the *CtDGAT2b* gene was transgenically introduced in the filamentous fungus following the standardized ATMT protocol. Putative fungal transformants were selected on hygromycin (200µg/ml) containing plates, and few stable transformants with either single copy or two copies genomic integrations of the transgene were obtained. After successful expression of the *CtDGAT2b* transgene, qualitative improvement of storage lipid and increase in the size of lipid bodies were observed in *Colletotricum* transformants with respect to the wild type strain as revealed through Nile red fluorescence staining assay. Moreover, difference in fatty acid profile with significant increase in the content of saturated fatty acids (C16:0 and C18:0) was also recorded in transformants compared to the wild type fungus. This could be due to the fact that the overexpression of *CtDGAT2b* gene, which has been isolated from the high stearate-rich *C. tropicalis* yeast strain, produces TAG with more saturated fatty acids as the CtDGAT2b enzyme has a natural tendency to pull saturated fatty acyl-CoAs. In fact, this preferential substrate specificity of CtDGAT2b has also been documented in our earlier study through heterologous expression in non-oleaginous yeast *Saccharomyces cerevisiae* [30].

From the quantitative estimation data on total lipid and neutral lipid fractions of transformants and wild type strain grown in standard and nutrient-stress conditions, it is evident that the overexpression of *CtDGAT2b* gene has prominant effect on enhancing the accumulation of storage lipid in transformed fungal lines. However, the four different transformed lines (Td#2, Td#9, Td#18 and Td#23) did not display much variation in accumulation of either total lipid or neutral lipid amongst them under all three conditions of growth (standard, nitrogen stress and phosphorus stress). Another interesting observation was noticed during growth of the wild type and transformant cells cultured for quantitative analysis of lipid. Although phenotypically (colony morphology) no differences were observed between wild type and transformant in plate culture, slight variation in growth morphology was found in liquid culture. When cultivated during standard growth condition or nutrient stress condition, wild type *Colletotrichum* cells usually grow by forming small aggregates or pellet-like structures and the culture is viscous. On the contrary, when grow in similar condition, all four transformed fungal lines produce less pellet and form cake-like morphology (data not shown), suggesting that the CtDGAT2b overexpression might have slight influence in cell physiology. As a consequence of this differential behavior, growth rate and biomass formation of the wild type and transformant demonstrated discripencies even when they were grown in similar conditions. Therefore, to further validate the comparison of lipid titers between the wild type and transformants of *Colletotrichum*, a model-based optimization of growth parameters was carried out to maximize lipid productivity in transformed fungal lines along with the wild type cells. A bioprocess optimization protocol has been established using ANN genetic algorithm, where 30 well distributed statistical data points were set with the help of CCD based on four critical parameters influencing lipid productivity in *Colletotricum* fungus such as temperature, pH, carbon: nitrogen (C:N) ratio and carbon: phosphorus (C:P) ratio according to our previous study [10].

RETRACTED

We have found that the wild type fungus can produce about 7.8±0.6 g/l of total lipid under nutrient (either nitrogen or phosphorus) stress condition, which is ∼1.6-fold more than the lipid titer (4.8±0.1 g/l) at standard growth condition. However, after model-based optimization of culture conditions, the wild type strain produces 9.1±0.8 g/l of total lipid i.e., ∼1.9-fold higher lipid titer without imposition of any nutrient stress (Figure 4). On the contrary, while the transformants at standard growth condition yield ∼1.7-fold more total lipid compared to the wild type (4.8±0.1 g/l increases to 8.1±0.2 g/l), optimization of culture conditions further increases the lipid titer upto 14.1±0.5 g/l or ∼1.7-fold higher in transformants (Figure 4). Taken together, ∼2.9-fold greater lipid titer over the wild type has been achieved in transformed *Colletotrichum* fungus following model-based optimization of culture condition and without any nutrient stress (Figure 4). Therefore, it is evident from the present study that not only biochemical engineering (nutrient stress) but the metabolic engineering of fungus using suitable gene together with bioprocess optimization could be an effective combined strategy to increase the storage lipid productivity. Critical analysis of our experimental data (Table 3) reveals that the lipid content in the transformed *Colletotrichum* is ∼1.9-fold higher under standard growth condition, and ∼2.2-fold more after model-based optimization of culture conditions as compared to the wild type strain grown at standard condition. In a previous report, the fungal genes coding for mailc enzyme from *Mucor circinelloides* (malEMt) and *Mortierella alpine* (malEMc) were overexpressed in *M. circinelloides*, which resulted 2.5- and 2.4-fold higher lipid content in the transformed malEMt and malEMc strains, respectively [22]. A recent report has documented 4-fold increase in lipid content compared to wild type through overexpression of *DGA1* gene (encoding for a type-1 DGAT) in *Yerrowia lipolytica* oleaginous yeast [43]. In the same organism, increased lipid content of 2-fold over control was observed after overexpression of acetyl-CoA carboxylase (ACC1) gene. Moreover, when both the genes (*ACC1+DGA1*) were overexpressed a lipid content of 4.9-fold was recorded in the same study. This ‘push-and-pull’ strategy can achieve large flux towards lipid accumulation with less feedback regulation as it maintain a balance between upstream and downstream metabolite formation pathway.

RETRACTED

**Figure 4:** Schematic representation of changes in lipid titer in the wild type and transformed *Colletotrichum* fungus after adopting different strategies.

## Conclusions

We have genetically modified an oleaginous filamentous endophytic fungus *Colletotrichum* sp. DM06 with the introduction of heterologous *CtDGAT2b* gene, which encodes a highly efficient version of DGAT enzyme responsible for enhanced TAG accumulation in rhizospheris yeast *C. tropicalis* SY005. Our laboratory-standardized method of *A. tumefacience*-mediated transformation was carried out to develop several independent transformed lines of *Colletotrichum*. Four stable transformants were investigated for the expression of *CtDGAT2b* transgene, qualitative assay and quantitative estimation of total lipid as well as neutral lipid. One of the stable transformants having single copy CtDGAT2b transgene in the fungal genome was further examined for the fatty acid profile of the total lipid and subjected to model-based bioprocess optimization for enhancement of lipid titer. Functional expression of CtDGAT2b successfully increases storage lipid titer as well as lipid content in genetically modified *Colletotrichum* with fatty acid profile being altered towards more palmitate and stearate. Prediction-based bioprocess optimization has been carried out to find the appropriate culturing conditions for lipid accumulation in both the wild type and transformed *Colletotrichum*. The lipid accumulation ability has been tested at optimum state of growth, and a net increase to 2.9-fold lipid titer over the wild type has been achieved due to genetic transformation of *Colletotrichum* sp. DM06 with the *CtDGAT2b* gene, which was not possible only by applying biochemical stress. To our knowledge, this is the first report to document genetic engineering coupled with model-based bioprocess optimization in an endophytic filamentous fungus for the enhancement of lipid productivity. In future such kind of genetic or metabolic engineering approach with important rate-limiting enzymes or critical transcription factors of lipid biosynthesis pathway along with the optimization of culture condition could further increase the lipid accumulation ability of oleaginous fungi or other microorganisms.

RETRACTED

## Supporting Information

Table S1 **Primers used in this study.**
(DOC)

Table S2 **Central composite design (CCD) of statistically distributed 30 different conditions based on four growth parameter.**
(DOC)

Table S3 **Experimentally determined biomass and lipid titers of the wild type** ***Colletotrichum*** **sp. grown in 30 different conditions.**
(DOC)

Table S4 **Experimentally determined biomass and lipid titers of transformed** ***Colletotrichum*** **sp. grown in 30 different conditions.**
(DOC)

Table S5 **Predicted and experimentally determined biomass and lipid titers of the wild type** ***Colletotrichum*** **sp. grown in 30 different conditions.**
(DOC)

Table S6 **Predicted and experimentally determined biomass and lipid titers of the transformed** ***Colletotrichum*** **sp. grown in 30 different conditions.**
(DOC)

Table S7 **Regression correlation coefficient (R^2^) between ANN-simulated values and experimental values of lipid titer in the wild type and transformed** ***Colletotrichum*** **sp.**
(DOC)
